RETRACTED

# Clinical Evaluation and Exploration of Mechanisms for Modified Xiebai Powder or Modified Xiebai Powder Combined with Western Medicine in the Treatment of Pneumonia

**DOI:** 10.1155/2022/2287470

**Published:** 2022-10-11

**Authors:** Qingling Zhang, Yuqi Zong, Lizhen Yang, Kunran Wang, Yan Wang

**Affiliations:** ^1^Post-Graduate Institute, Heilongjiang University of Chinese Medicine, Harbin 150040, Heilongjiang, China; ^2^Institute of Pharmaceutical & Food Engineering, Shanxi University of Chinese Medicine, Jinzhong 030619, Shanxi, China

## Abstract

**Objective:**

To systematically evaluate the clinical efficacy of modified Xiebai Powder or modified Xiebai Powder combined with Western medicine in the treatment of pneumonia and explore its potential mechanism of action.

**Methods:**

Meta-analysis was used to screen the eligible literature on randomized controlled trials (RCTs) about Xiebai Powder in the treatment of pneumonia, and Review Manager 5.3 software was used for statistical analysis of the data. Based on the results of the meta-analysis, the active ingredients in Xiebai Powder and their therapeutic targets, disease-related targets, and intersection targets were screened using methods of network pharmacology, and their biological processes and key signaling pathways were analyzed using bioinformatics tools. Molecular docking was carried out to verify and predict the mechanisms for Xiebai Powder combined with Western medicine in the treatment of pneumonia.

**Results:**

A total of 16 papers were screened out, with a total of 1,465 patients. The results of the meta-analysis showed that modified Xiebai Powder or modified Xiebai Powder combined with Western medicine were superior to conventional Western medicine in terms of clinical efficacy, shortening the disappearance time of symptoms (body temperature, cough, and pulmonary rales) and reducing the level of C-reactive protein, and the incidence of adverse reactions was significantly reduced. A total of 40 active ingredients in Xiebai Powder and 285 therapeutic targets of Xiebai Powder combined with azithromycin after deduplication were screened out from the database. KEGG enrichment analysis showed that Xiebai Powder combined with azithromycin might play a role in the treatment of pneumonia through the IL-17 signaling pathway, tumor necrosis factor signaling pathway, C-type lectin receptor signaling pathway, Toll-like receptor signaling pathway, and HIF-1 signaling pathway.

**Conclusions:**

Modified Xiebai Powder or modified Xiebai Powder combined with azithromycin has better effects in treating pneumonia, and modified Xiebai Powder combined with azithromycin may play a role in treating pneumonia through several pathways such as the IL-17 signaling pathway.

RETRACTED

## 1. Introduction

Pneumonia is an acute inflammation of the lower respiratory tract and lung parenchyma, and the main clinical symptoms are fever, cough, and shortness of breath [1]. It is usually caused by bacterial and viral infections [2], which is common in children, the elderly, and people with poor immune functions. The high incidence and high mortality of pneumonia worldwide pose a great threat to human lives. There are many adverse reactions and drug resistance in the treatment of pneumonia with antibiotics, which are widely used in clinics at present. For example, azithromycin preparation is widely used in clinic and is one of the mainstream antibacterial drugs for community-acquired pneumonia (CAP) in children. Aiming at the minimum applicable age for azithromycin treatment and according to the guidelines for the management of community-acquired pneumonia in children (revised in 2013), the efficacy and safety of azithromycin have not been established for children younger than six months with CAP, so it should be used with caution [3]. Increasing numbers of reports have shown that the TCM treatment of pneumonia has the advantages of lower incidence of adverse reactions and outstanding clinical efficacy.

Xiebai Powder is a classic prescription that comes from *Key to Therapeutics of Children's Diseases*, written by Qianyi in the Northern Song Dynasty. *Key to Therapeutics of Children's Disease*s an early monograph on syndrome differentiation and treatment of pediatric diseases in China. It is also the first existing pediatric book preserved in the form of the original book in the world. It is available in Japan and some other countries and has a wide range of influence [4]. Xiebai Powder contains four kinds of herbs, including Cortex Mori, Cortex Lycii, licorice root, and japonica rice, which have the functions of clearing away lung heat, relieving cough, and relieving asthma [5]. In Xiebai Powder, the amount of Cortex Mori and Cortex Lycii is one *liang* each, licorice is one *qian*, and the amount of japonica rice is a *zuo* [6]. Cortex Mori, Cortex Lycii, and licorice root are three plant-derived traditional Chinese medicines in Xiebai Powder. They are specified and recorded in the Chinese Pharmacopoeia and the Japanese Pharmacopoeia, and their sources, uses, and active ingredients are specified [7]. Modified prescription of Xiebai Powder is more widely used in the modern clinic for the treatment of pneumonia and other pulmonary diseases [8], but the current evidence-based basis is insufficient, and the mechanism of action is not clear. The clinical efficacy of modified Xiebai Powder or modified Xiebai Powder combined with western medicine in treating pneumonia was evaluated in this study by collecting published literature of RCTs. Based on meta-analysis, the potential mechanisms for Xiebai Powder in treating pneumonia was analyzed using network pharmacology to provide a basis for subsequent studies.

RETRACTED

## 2. Materials and Methods

### 2.1. Meta-Analysis

#### 2.1.1. Inclusion Criteria

For RCTs published in both Chinese and English, adult patients in the study should meet the diagnostic criteria published in the Chinese Journal of Tuberculosis and Respiratory Diseases in 2016 [9], and children should meet the diagnostic criteria published in the Chinese Journal of Pediatrics in 2013 [3].

#### 2.1.2. Exclusion Criteria

Duplicate publications, unobtainable literature, literature with incomplete or erroneous information, reviews, medical records, experience summaries, animal experiments, nonrandomized controlled experiments, inconsistent experimental designs, and patients with other comorbidities (such as heart failure) were excluded.

#### 2.1.3. Primary Outcomes

Clinical efficacy, body temperature recovery time, cough disappearance time, pulmonary rales disappearance time, and C-reactive protein level were used as primary outcomes.

#### 2.1.4. Interventions

Patients in the control group were treated with Western medicine. Patients in the experimental group were treated with modified Xiebai Powder or modified Xiebai Powder combined with Western medicine.

#### 2.1.5. Strategies for Literature Retrieval

The Chinese retrieval platforms used include CNKI, VIP, and Wanfang. The English databases used include PubMed, Cochrane Library, and Science Direct. Relevant Chinese and English literature from the establishment of the databases to January 2022 were obtained. The keywords of English and Chinese retrieval were “Xiebai Powder (泻白散),” “pneumonia (肺炎),” etc.

#### 2.1.6. Data Extraction and Quality Assessment

After obtaining the eligible literature, relevant information such as title, first author, publication time, gender of patients, sample size, name of the disease, classification of disease, treatment measures, and outcomes were extracted. RCTs were reviewed using the Cochrane Handbook for random sequence generation, allocation concealment, blinding (subjects, experimenters, and evaluators), completeness of outcome data, selective reporting, and other biases [10]. The assessment of “low risk,” “high risk,” and “unclear risk” were given according to the specific content of the literature.

#### 2.1.7. Data Statistics and Analysis

Review Manager 5.3 software was used for statistical analysis. Enumeration data were analyzed with an odds ratio (OR), mean difference (MD) for measurement data, and 95% confidence interval (CI) for efficacy analysis and statistics. *P* ≤ 0.05 indicated a statistically significant difference. The Chi-square test was used to evaluate statistical heterogeneity between studies. *P*°≥0.1 and *I*^2^°≤°50% indicated no heterogeneity, and analysis was performed using a fixed-effects model; otherwise, a random-effects model was used, combined with subgroup analysis or sensitivity analysis to find the source of heterogeneity.

RETRACTED

### 2.2. Network Pharmacological Study on Xiebai Powder Combined with Western Medicine in the Treatment of Pneumonia

#### 2.2.1. Screening of Active Ingredients of Xiebai Powder

According to the published literature [11, 12], and taking “Cortex Mori,” “Cortex Lycii,” and “licorice root” as the keywords, the chemical ingredients of the three herbs were retrieved using the TCMSP database (https://old.tcmsp-e.com/tcmsp.php), and the active ingredients of the drugs were screened according to the oral bioavailability (OB) ≥ 30% and the drug‐likeness (DL) ≥ 0.18.

#### 2.2.2. Acquisition of Therapeutic Targets of Active Ingredients of Xiebai Powder and Azithromycin and Disease-Related Targets

The active ingredients of Xiebai Powder were obtained from the TCMSP database, and the names of protein targets were converted to gene names using the UniProt database. Azithromycin was retrieved in the TTD database, and the canonical SMILES structure was imported into the Swiss Target Prediction database and the SEA database to obtain the therapeutic targets. The Gene Cards database was used to search the keyword “pneumonia” to obtain pneumonia-related targets, and the DisGeNET database and the TTD database were used to complement pneumonia-related targets.

#### 2.2.3. Construction of Protein-Protein Interaction (PPI) Network and Acquisition of Key Targets

The intersection targets of active ingredients of Xiebai Powder combined with azithromycin and pneumonia were identified using the Venny2.1 online tool and imported into the STRING database for PPI analysis. Limiting the species to “Homo sapiens,” a PPI network was constructed. The PPI network data was imported into Cytoscape 3.9.1 software and topologically analyzed using the Analyze Network function. The medians of degree centrality, closeness centrality (CC), and betweenness centrality (BC) were taken as the chi values to screen key targets.

#### 2.2.4. KEGG Pathway Enrichment Analysis

The intersection targets screened in Section 2.2.3 were imported into the DAVID database for KEGG pathway enrichment analysis, and the results were visualized using the bioinformatics data analysis platform.

RETRACTED

#### 2.2.5. Molecular Docking

Key targets with top degree values were selected and input into the PDB database. Their 3D structures were downloaded and saved in the PDB format, and water molecules and other ligands were removed using PyMol software. The top eight active ingredients in Xiebai Powder, according to the degree values, and the SDF format files of the active ingredients were downloaded from the PubChem database and imported into OpenBabel to be converted into PDB format. Proteins were hydrogenated using AutoDock. The Grid Box in the Grid module was set, and the vina program was used to semiflexible dock targets (receptors) with chemical ingredients (ligands). The combinations with the lowest binding energy were selected and visualized using PyMol software.

## 3. Results

### 3.1. Meta-Analysis

#### 3.1.1. Literature Screening and the Basic Characteristics of Included Literature

A total of 138 related papers were retrieved, and 16 papers on RCTs were included according to the inclusion and exclusion criteria, with a total of 1465 patients, including 744 cases in the experimental group and 721 cases in the control group. The specific process of literature screening is shown in Figure 1. The basic characteristics of the 16 papers are shown in Table 1.

#### 3.1.2. Quality Assessment and Publication Bias Assessment of Included Literature

All RCTs were randomly grouped, of which two [13, 14] were grouped by a random number table and rated as “low risk; ” one [15] was grouped according to the order of admission and rated as “high risk; ” the remaining 13 RCTs were rated as “high risk.” All RCTs without allocation concealment and blinding were rated as “unclear risk.” All RCTs with precise outcomes were rated as “low risk.” None of the RCTs mentioned selective reporting, and all RCTs were rated as “unclear risk.” All RCTs with unclear other biases were rated as “unclear risk.” The specific information is shown in Figure 2.

#### 3.1.3. Meta-Analysis of Each Primary Outcome

*(1) Clinical Efficacy*. All studies [13–28] reported clinical efficacy. The heterogeneity testing result showed no heterogeneity (*P*° = 0.89, *I*^2^° = °0%), and a fixed-effects model was used for analysis. The results showed that the clinical efficacy in the experimental group (modified Xiebai Powder or modified Xiebai Powder combined with Western medicine treatment) was better than that in the control group (conventional Western medicine treatment) (OR° = 5.42, 95% CI (3.72, 7.88), *P*°<0.00001; Figure 3).

*(2) Body Temperature Recovery Time*. A total of five papers [13, 17, 18, 24, 25] reported the body temperature recovery time in patients with pneumonia, and the heterogeneity testing result showed great heterogeneity (*P*°<0.00001, *I*^2^° = °97%). Subgroup analysis was performed according to whether the disease was clearly classified. The heterogeneity testing result of the three studies with unknown disease classification was *P*°<0.00001 and *I*^2^° = °96%, and the heterogeneity testing result of the two studies with well-defined disease classification was *P*°<0.00001 and *I*^2^° = °99%, indicating that disease classification was not the source of heterogeneity in this outcome. It is found by sensitivity analysis that the heterogeneity came from three studies [18, 24, 25], which were removed, and the remaining two studies [13, 17] were retested without heterogeneity (*P*° = 0.75, *I*^2^° = °0%) and analyzed by a fixed-effects model. The results showed that the body temperature recovery time in the experimental group (modified Xiebai Powder combined with conventional Western medicine treatment) was shorter than that in the control group (conventional Western medicine treatment) (*MD*° = °−2.06, 95% CI (-2.31, -1.82), *P*°<0.00001; Figure 4). A descriptive analysis was conducted for three excluded studies, in which the effects of modified Xiebai Powder combined with conventional Western medicine treatment on shortening the body temperature recovery time in patients with pneumonia were compared. Meta-analysis results were as follows: MD° = °−1.12, 95% CI (-1.34, -0.90), *P*°<0.00001; MD° = °−0.47, 95% CI (-0.61, -0.33), *P*°<0.00001; MD° = °−0.79, 95% CI (-0.87, -0.71), *P*°<0.00001. By analyzing and comparing the results, it was found that modified Xiebai Powder combined with conventional Western medicine had a better therapeutic effect than conventional Western medicine alone.

*(3) Cough Disappearance Time*. Five papers [13, 17, 18, 20, 25] reported the cough disappearance time in patients with pneumonia, and the heterogeneity testing result showed great heterogeneity (*P*°<0.00001, *I*^2^° = °97%). Subgroup analysis was performed according to whether the disease was clearly classified. The heterogeneity testing result of the two studies with unknown disease classification was *P*°<0.00001 and *I*^2^° = °97%, and the heterogeneity testing result of the three studies with well-defined disease classification was *P*°<0.00001 and *I*^2^° = °36%, indicating that disease classification was not the source of heterogeneity in this outcome. Sensitivity analysis showed that the heterogeneity came from three studies [13, 17, 18], which were removed, and the remaining two studies [20, 25] were retested without heterogeneity (*P*° = 0.89, *I*^2^° = °0%) and analyzed by a fixed-effects model. The results showed that the elimination of cough in the experimental group was more effective than that in the control group (MD° = °−3.18, 95% CI (-3.78, -2.57), *P*°<0.00001; Figure 5). A descriptive analysis was conducted for the three excluded studies, in which the effects of modified Xiebai Powder combined with conventional Western medicine treatment on shortening the cough disappearance time in patients with pneumonia were compared. Meta-analysis results were as follows: MD° = °−1.89, 95% CI (-2.18, -1.60), *P*°<0.00001; MD° = °−5.60, 95% CI (-6.14, -5.06), *P*°<0.00001; MD° = °−2.20, 95% CI (-2.47, -1.93), *P*°<0.00001. By analyzing and comparing the results, it was found that modified Xiebai Powder combined with conventional Western medicine had a better therapeutic effect than conventional Western medicine.

*(4) Pulmonary Rales Disappearance Time*. A total of five papers [13, 17, 18, 24, 25] reported the pulmonary rales disappearance time in patients with pneumonia, and the heterogeneity testing result showed heterogeneity (*P*° = 0.001, *I*^2^° = °77%). Subgroup analysis was performed according to whether the disease was clearly classified. The heterogeneity testing result of the three studies with unknown disease classification was *P*°<0.00001 and *I*^2^° = °82%, and the heterogeneity testing result of the two studies with well-defined disease classification was *P*°<0.00001 and *I*^2^° = °72%, indicating that disease classification was not the source of heterogeneity in this outcome. Sensitivity analysis showed that the heterogeneity came from two studies [17, 24], which were removed, and the remaining three studies [13, 18, 25] were retested with small heterogeneity (*P*° = 0.15, *I*^2^° = °47%) and analyzed by a fixed-effects model. The results showed that the elimination of pulmonary rales in the experimental group was more effective than that in the control group (MD = −2.09, 95% CI (-2.30, -1.88), *P* < 0.00001; Figure 6). A descriptive analysis was conducted for the two excluded studies, in which the effects of modified Xiebai Powder combined with conventional Western medicine treatment on shortening the pulmonary rales disappearance time in patients with pneumonia were compared. Meta-analysis results were as follows: MD = −3.57, 95% CI (-4.72, -2.42), *P* < 0.00001; MD = −1.70, 95% CI (-1.93, -1.47), *P* < 0.00001. By analyzing and comparing the results, it was found that modified Xiebai Powder combined with conventional Western medicine had a better therapeutic effect than conventional Western medicine.

*(5) C-Reactive Protein (CRP)*. A total of three papers [16, 19, 25] analyzed the level of C-reactive protein in patients with pneumonia, and the heterogeneity testing result showed great heterogeneity (*P*°<0.00001, *I*^2^° = °100%). Sensitivity analysis found that the heterogeneity came from 1 study [25], which was removed, and the remaining two studies [16, 19] were retested with small heterogeneity (*P*° = 0.18, *I*^2^° = °43%) and analyzed by a fixed-effects model. The results showed that the reduction of CRP level in the experimental group was more effective than that in the control group (MD = −3.05, 95% CI (-4.24, -1.85), *P* < 0.00001; Figure 7). A descriptive analysis was conducted for one excluded study, in which the effects of modified Xiebai Powder combined with conventional Western medicine treatment on reducing CRP levels were compared. Meta-analysis showed that the effect of reducing CRP levels in the experimental group was better than that in the control group (MD = −49.19, 95% CI (-52.16, -46.22), *P* < 0.00001).

RETRACTED

#### 3.1.4. Adverse Reactions

A total of three papers [13, 18, 24] mentioned the adverse reactions in patients, among which the incidence of adverse reactions was counted in three studies [13, 24], and one study [18] showed no adverse reactions in patients. The heterogeneity testing result exhibited no heterogeneity (*P*° = 0.84, *I*2° = °0%), and a fixed-effects model was used for analysis. The results showed that the incidence of adverse reactions in the experimental group (modified Xiebai Powder combined with conventional Western medicine treatment) was lower than that in the control group (conventional Western medicine treatment) (OR = 0.33, 95% CI (0.15, 0.69), *P* = 0.003; Figure 8).

#### 3.1.5. Publication Bias Analysis

Publication bias analysis was performed on clinical effective rates, and funnel plots were drawn to observe symmetry. The number of points on the left side of Figure 9 is 11, and the number of points on the right side is 5. There was a significant difference in the number distribution of points between both sides, indicating a certain publication bias (Figure 9).

#### 3.1.6. Sensitivity Analysis

Sensitivity analysis was performed on the included literature, and descriptive analysis was performed on the results. The pooled effect size of clinical effective rates in the 16 studies was excluded. The results showed no qualitative change in the pooled effect size, and the results of this study were relatively stable.

### 3.2. Network Pharmacology

#### 3.2.1. Screening of Active Ingredients in Xiebai Powder and Pneumonia-Related Targets

There were 40 active ingredients with 235 therapeutic targets in Xiebai Powder, including ten in Cortex Mori, ten in Cortex Lycii, 16 in licorice root, and four repetitive ingredients. Azithromycin (drug ID: D03HJK, molecular formula: C_38_H_72_N_2_O_12_) had 55 target genes. Xiebai Powder combined with azithromycin had 285 therapeutic targets after deduplication. A total of 1359 pneumonia-related targets were retrieved through the Gene Cards database, 1032 through the DisGeNET database, and 17 through the TTD database. After deduplication, 1926 pneumonia-related targets were collected (Table 2).

RETRACTED

#### 3.2.2. Construction of the Drug-Active Ingredient-Target Network

The “drug-active ingredient-target” visualized network is shown in Figure 10. According to the degree value, the top active ingredients were *β*-sitosterol, quercetin, kaempferol, naringenin, acacetin, isorhamnetin, etc., as shown in Table 3.

#### 3.2.3. Construction of PPI Network and Screening of Key Targets

After using the Venny 2.1 online tool to intersect the targets of active ingredients in Xiebai Powder and the pneumonia-related targets, a total of 129 common targets were obtained, as shown in Figure 11. The common targets were input into the STRING database to obtain the PPI network, which was processed by Cytoscape 3.9.1 software. There were 129 nodes and 2783 edges in the network (Figure 12). After topological analysis, the chi values of degree ≥ 85, CC ≥ 0.744, and BC ≥ 200.368 were selected as the screening conditions, and the targets that met the above three chi values were selected as key targets, mainly including TNF, IL-6, ALB, AKT1, IL-1*Β*, TP53, CASP3, PTGS2, JUN, and STAT3 (Table 4).

#### 3.2.4. Enrichment Analysis

A total of 169 signaling pathways were obtained through KEGG pathway enrichment analysis (*P* < 0.05), and the top 20, according to the *P* value ranking, were plotted (Figure 13). Xiebai Powder combined with azithromycin may play a role in the treatment of pneumonia through the IL-17 signaling pathway, tumor necrosis factor signaling pathway, c-type lectin receptor signaling pathway, Toll-like receptor signaling pathway, and HIF-1 signaling pathway.

#### 3.2.5. Molecular Docking

The active ingredients and key targets with high degree values were selected, and AutoDock software was used for molecular docking. The results are shown in Table 5. All active ingredients and key targets can spontaneously bind (the binding free energy was less than 0 kJ·mol^−1^). The docking results were visualized by PyMol software, partially shown in Figure 14.

## 4. Discussion

During the analysis of this study, a total of 138 papers were read, and only 16 papers in Chinese were eligible for this systematic review and meta-analysis, with a total of 1,465 patients. Clinical efficacy, body temperature recovery time, cough disappearance time, pulmonary rales' disappearance time, and C-reactive protein level were selected as primary outcomes. Meta-analysis results showed that all the outcomes were statistically significant, indicating that modified Xiebai Powder or modified Xiebai Powder combined with conventional Western medicine treatment had better effects than conventional Western medicine treatment.

RETRACTED

Due to the limitation of the overall level and quantity of the literature included in this study, more high-quality literature should be included in the follow-up to further verify the analysis results. The outcomes in the included literature were mainly clinical efficiency and clinical manifestation, and less attention was paid to the changes in vital signs (respiratory rate, heart rate, systolic blood pressure, etc.) [29], procalcitonin [30], and T cell population [30, 31]. It is suggested to add relevant outcomes to related RCTs in the future to improve the accuracy of clinical efficacy evaluation and quality of evidence.

The network pharmacological analysis showed that the main active ingredients in Xiebai Powder in the treatment of pneumonia involved *β*-sitosterol, quercetin, kaempferol, naringenin, isorhamnetin, and other compounds. Among them, *β*-sitosterol is a phytosterol, and the others are flavonoids. *β*-Sitosterol can inhibit proinflammatory cytokines such as TNF-*α* and IL-6. A number of in vitro and in vivo experiments have shown that quercetin has anti-inflammatory activity and can also inhibit apoptosis and repair damaged lung tissue by inhibiting the growth and metastasis of lung cancer cells [32]. Kaempferol has the effects of anti-inflammation, antioxidation, and inhibiting apoptosis. Both naringenin and isorhamnetin have anti-inflammatory activities and can significantly reduce the levels of proinflammatory cytokines in serum and lung tissue [33]. It can be seen that the above active ingredients play important roles in the treatment of pneumonia.

Results of network pharmacology and molecular docking show that beta-sitosterol can inhibit the proinflammatory cytokines TNF-*α* and IL-6. Beta-sitosterol is one of the effective components of TCM. Maxing Shigan Decoction comes from the treatise on *Shang Han Lun* and is composed of Ephedrae herba, armeniacae semen amarum, gypsum fibrosum, and Glycrrhizae Radix et Rhizoma. Among the four TCM, Ephedrae herba, armeniacae semen amarum, and Glycrrhizae Radix et Rhizoma all contain *β*-sitosterol [34–36]. Maxing Shigan decoction combined with azithromycin in the treatment of mycoplasma pneumonia in children is more effective than azithromycin alone [37].

Qianjin Weijing decoction is derived from *Jin Kui Yao Lue*. It is composed of Phragmitis rhizome, Coicis Semen, coix seed, and Persicae Semen. These four TCMs all contain human *β*-sitosterol [38–40]. Qianjin Weijing decoction combined with azithromycin in the treatment of Mycoplasma pneumoniae pneumonia in children can effectively alleviate clinical symptoms [41]. From the perspective of traditional Chinese medicine, Xiebai powder, Maxing Shigan Decoction, and QianjinWeijing decoction have different functions. Xiebai powder is mainly used for asthma and cough, skin steaming, and heat, especially the illness worsens in the morning.

RETRACTED

The key targets of Xiebai Powder combined with azithromycin in the treatment of pneumonia were mainly TNF, IL-6, ALB, AKT1, IL-1*Β*, TP53, CASP3, PTGS2, JUN, STAT3, etc. Among them, both TNF and IL-6 are inflammatory factors. A study showed that the levels of TNF-*α* and IL-6 in patients with pneumonia were significantly increased, indicating that TNF-*α* and IL-6 genes were involved in the onset of pneumonia [42]. ALB is highly correlated with acute lung injury and is a predictor of disease severity [43]. TP53 is a tumor suppressor gene involved in the regulation of the cell cycle and apoptosis, and its overexpression can promote cancer [44]. IL-1*Β* has been found to be a targeted treatment for COVID-19 [45]. STAT3 protein is involved in the transcription of inflammatory factors after entering the nucleus. The inhibition of the activation of transcription factor AP-1 can reduce the proinflammatory response induced by IL-1*Β*. It is speculated that the expression of the abovementioned transcription factor proteins is closely related to inhibiting the occurrence of the inflammatory response [46].

The KEGG analysis showed that Xiebai Powder might play a role in the treatment of pneumonia through the hepatitis B-induced signaling pathway, cancer signaling pathway, toxoplasmosis-induced signaling pathway, Toll-like receptor signaling pathway, tumor necrosis factor signaling pathway, and pertussis-induced signaling pathway. The KEGG analysis showed that azithromycin might play a role in the treatment of pneumonia through the IL-17 signaling pathway, NOD-like receptor signaling pathway, Toll-like receptor signaling pathway, TNF signaling pathway, and PI3K-Akt signaling pathway.

The KEGG enrichment pathways of Xiebai Powder combined with azithromycin mainly involved the IL-17 signaling pathway, tumor necrosis factor signaling pathway, c-type lectin receptor signaling pathway, Toll-like receptor signaling pathway, and HIF-1 signaling pathway. The IL-17 signaling pathway is associated with the occurrence and development of pneumonia-induced sepsis. In addition, the upregulation of upstream and downstream molecules in the IL-17 signaling pathway indicates the activation of the IL-17 signaling pathway, which can promote apoptosis in pneumonia-induced sepsis [47]. Excessive TNF-*α* in the tumor necrosis factor signaling pathway can not only lead to abnormal pathways but also promote inflammatory factors such as IL-1 and IL-8, stimulate the body's inflammatory responses, or even cause inflammatory chain reactions [48]. The Toll-like receptor signaling pathway transmits signals into cells by recognizing lipopolysaccharide and finally activates inflammatory factors such as TNF to mediate the inflammatory response in diseased tissues [49].

RETRACTED

The main KEGG pathways of azithromycin in pediatric pneumonia are the IL-17 signaling pathway, NOD-like receptor signaling pathway, Toll-like receptor signaling pathway, TNF signaling pathway, and PI3K-Akt signaling pathway. NOD-like receptors can mediate inflammatory responses, activate NF-B p65 and p38 MAPK signaling pathways, and lead to the production of inflammatory factors [50]. A NOD-like receptor signaling pathway is the main difference between the action pathway of Xiebai Powder combined with azithromycin and that of azithromycin.

## 5. Conclusions

In this study, meta-analysis combined with network pharmacology was used to evaluate Xiebai Powder in the treatment of pneumonia systematically and to predict its potential mechanism of action. In terms of clinical efficacy, body temperature recovery time, cough disappearance time, pulmonary rales' disappearance time, and C-reactive protein reduction, the experimental group was superior to the control group, with a lower incidence of adverse reactions.

Also, the mechanism for Xiebai Powder combined with azithromycin in the treatment of pneumonia was analyzed using network pharmacology. Due to the complexity of chemical ingredients and targets of TCM and their effects on the human body, further studies are needed to provide more evidence. Based on the potential pathways obtained through meta-analysis and network pharmacological studies, the next step will be to obtain key pathways based on cell level or animal experiments to study the mechanisms of Xibai Powder in the treatment of pediatric pneumonia.

Overall, the analysis results are credible. More high-quality papers will be included in the follow-up to verify the analysis results further. Considering dynamic changes in pneumonia studies, in future research, other relevant outcomes such as changes in vital signs (respiratory rate, heart rate, systolic blood pressure, etc.), procalcitonin (PCT), and T cell population will be added to improve the accuracy of clinical efficacy evaluation further and enhance the quality of evidence.

## Figures and Tables

**Figure 1:** The flow chart of literature screening for meta-analysis.

RETRACTED

**Figure 2:** (a) Overall risk of bias graph. (b) Detailed risk of bias summary.

**Figure 3:** Meta-analysis forest plot of clinical efficacy.

**Figure 4:** Meta-analysis forest plot of body temperature recovery time.

**Figure 5:** Meta-analysis forest plot of cough disappearance time.

**Figure 6:** Meta-analysis forest plot of pulmonary rales' disappearance time.

**Figure 7:** Meta-analysis forest plot of C-reactive protein.

**Figure 8:** Meta-analysis forest plot of adverse reactions.

**Figure 9:** Publication bias funnel plot.

**Figure 10:** Drug-ingredients-targets diagram. Note: the orange diamonds represent the target genes of the ingredients; the yellow circles represent the three herbs; the hexagons represent the ingredients contained; the octagons represent the common ingredients. SBP: Cortex Mori; DGP: Cortex Lycii; GC: licorice root; AQMS: azithromycin.

**Figure 11:** Common target Venny diagram.

**Figure 12:** PPI network diagram of Xiebai Powder combined with azithromycin.

**Figure 13:** Bubble diagram of KEGG pathway enrichment analysis.

**Figure 14:** Visualization of molecular docking results (part): (a) quercetin-tp53, (b) kaempferol-tp53, (c) naringenin-IL-1*Β*, (d) acacetin-IL6, (e) Inermine-ALB, and (f) isorhamnetin-TNF.

**Table 1:** Essential features of the included literature.

No.	Eligible studies	Sample size (T/C)	Sexuality (M/F)	Intervention measures		Disease	Disease classification	Observed indexes
				T	C			
1	Sun et al. [16]	70 (35/35)	T: 21/14 C: 20/15	Modified Xiebai Power+conventional Western medicine treatment	Conventional Western medicine treatment	Senile pneumonia	Qi and Yin deficiency type	①⑥⑦⑧
2	Xu et al. [13]	106 (53/53)	T: 31/22 C: 30/23	Modified Xiebai Power+conventional Western medicine treatment	Conventional Western medicine treatment	Mycoplasmal pneumonia in children	Yin deficiency due to lung heat	①②③⑤
3	Wei [17]	200 (100/100)	T: 49/51 C: 58/42	Modified Xiebai Power+conventional Western medicine treatment	Conventional Western medicine treatment	Pediatric pneumonia	Unknown	①②③⑤
4	Chen et al. [14]	72 (36/36)	T: 22/14 C: 24/12	Xiebai Power modified recipe+conventional rehabilitation comprehensive therapy	Conventional comprehensive rehabilitation therapy	Severe pneumonia	Lung phlegm heat syndrome	①⑨
5	Wang et al. [18]	64 (32/32)	T: 18/14 C: 17/15	Xiebai Power modified recipe combined with traditional Chinese medicine iontophoresis+conventional Western medicine treatment	Conventional Western medicine treatment	Pediatric pneumonia	Wind-heat and closed lung type	①②③⑤
6	Liu [19]	50 (25/25)	T: 15/10 C: 14/11	Modified Xiebai Power+conventional Western medicine treatment	Conventional Western medicine treatment	Community-acquired pneumonia	Unknown	①④⑥⑦⑩
7	Guan [20]	72 (36/36)	T: 18/18 C: 20/16	Xiebai Power addition and subtraction formula	Conventional Western medicine treatment	Chronic cough after mycoplasma pneumonia in children	Lung heat yin deficiency type	①③④
8	Ding and Wang [21]	64 (32/32)	T: 18/14 C: 17/15	Modified Xiebai Power+conventional Western medicine treatment	Conventional Western medicine treatment	Mycoplasmal pneumonia in children	Phlegm-heat closed lung type	①
9	Fu [22]	66 (36/30)	T: 21/15 C: 20/10	Modified Xiebai Power+conventional Western medicine treatment	Conventional Western medicine treatment	Interstitial pneumonia in children	Unknown	①
10	Liang et al. [15]	137 (77/60)	T: 52/25 C: 42/18	Modified Xiebai Power+conventional Western medicine treatment	Conventional Western medicine treatment	Senile pneumonia	Unknown	①
11	Yang [23]	158 (79/79)	T: 48/31 C: 44/35	Modified Xiebai Power+conventional Western medicine treatment	Conventional Western medicine treatment	Senile pneumonia	Unknown	①
12	Han [24]	90 (45/45)	T: 25/20 C: 27/18	Modified Xiebai Power+conventional Western medicine treatment	Conventional Western medicine treatment	Mycoplasmal pneumonia in children	Unknown	①②④⑤⑪⑫⑬
13	Liu et al. [25]	60 (30/30)	33/27	Modified Xiebai Power+conventional Western medicine treatment	Conventional Western medicine treatment	Mycoplasmal pneumonia in children	Unknown	①②③ ⑤⑦⑧
14	Yu et al. [26]	88 (44/44)	52/36	Modified Xiebai Power+conventional Western medicine treatment	Conventional Western medicine treatment	Mycoplasmal pneumonia in children	Unknown	①
15	Li and Li [27]	120 (60/60)	64/56	Xiebai Power+conventional western medicine treatment	Conventional Western medicine treatment	Pneumonia	Unknown	①
16	Sun and Chang [28]	48 (24/24)	26/22	Modified Xiebai Power+conventional Western medicine treatment	Conventional Western medicine treatment	Mycoplasmal pneumonia in children	Unknown	①

T: test team; C: control group; M: male; F: female. ① Clinical efficacy. ② Body temperature recovery time. ③ Cough disappearance time. ④ Cough improvement time. ⑤ Time of pulmonary rale disappearance. ⑥ WBC. ⑦ CRP. ⑧ NEUR. ⑨ sTREM-1 and suPAR levels. ⑩ ESR. ⑪ IL-6. ⑫ IL-8. ⑬ TNF.

RETRACTED

**Table 2:** Basic biological information of Xiebai Powder combined with azithromycin.

Category	Herb	Number of effective components	Number of target genes
Xiebai Powder	Cortex Lycii	10	81
	Cortex Mori	10	177
	Licorice root	16	218
Western medicine	Azithromycin	1	55

**Table 3:** Top 10 active ingredients of Xiebai Powder for treating pneumonia.

MOL ID	Name	Source	OB (%)	DL	Degree
MOL000098	Quercetin	Morus alba, licorice	46.43	0.28	192
MOL000422	Kaempferol	Morus alba, licorice	41.88	0.24	42
MOL000358	Beta-sitosterol	Morus alba, Cortex Lycii	36.91	0.75	35
MOL001552	OIN	Cortex Lycii	45.97	0.19	26
MOL004328	Naringenin	Licorice	59.29	0.21	24
MOL001689	Acacetin	Cortex Lycii	34.97	0.24	23
MOL001484	Inermine	Licorice	75.18	0.54	17
MOL000354	Isorhamnetin	Licorice	49.60	0.31	15
MOL002565	Medicarpin	Licorice	49.22	0.33	12
MOL012681	Dimethyl (methylenedi-4,1-phenylene) biscarbamate	Morus alba	50.84	0.26	10

**Table 4:** Top 10 core target genes.

No.	Target	Degree	Betweenness	Closeness
1	TNF	109	702.4166	0.8707483
2	IL6	109	908.7839	0.8707483
3	ALB	109	984.4666	0.8707483
4	AKT1	107	822.7076	0.8590604
5	IL-1*Β*	102	513.9354	0.8311688
6	TP53	93	404.8256	0.7852761
7	CASP3	88	276.6789	0.7573965
8	PTGS2	87	274.6361	0.7485380
9	JUN	86	200.3681	0.7529412
10	STAT3	85	246.6801	0.7441860

**Table 5:** The docking results of core components and key target molecules.

Component	Binding free energy of active components to key targets (kJ·mol^−1^)					
	TNF	IL6	ALB	AKT1	IL-1*Β*	TP53
Quercetin	-6.0	-7.1	-7.0	-7.8	-7.0	-8.0
Kaempferol	-4.5	-4.5	-4.1	-4.8	-4.4	-5.5
Beta-sitosterol	-7.0	-4.5	-6.3	-9.4	-4.4	-5.5
OIN	-5.9	-6.0	-5.8	-7.6	-6.2	-6.4
Naringenin	-6.5	-6.5	-7.1	-9.3	-7.3	-7.6
Acacetin	-9.2	-7.9	-8.4	-11.8	-8.5	-9.8
Inermine	-7.1	-6.8	-6.5	-8.3	-7.2	-7.8
Isorhamnetin	-6.9	-6.7	-6.9	-9.1	-7.0	-7.4

## Data Availability

The data used to support the findings of this study are included within the article.
